# PD-L1 diagnostic tests: a systematic literature review of scoring algorithms and test-validation metrics

**DOI:** 10.1186/s13000-018-0689-9

**Published:** 2018-02-09

**Authors:** Margarita Udall, Maria Rizzo, Juliet Kenny, Jim Doherty, SueAnn Dahm, Paul Robbins, Eric Faulkner

**Affiliations:** 1 Pfizer Inc, New York, NY USA; 2 Evidera, Metro Building, 6th Floor, 1 Butterwick, London, W6 8DL UK

**Keywords:** Cancer, Immunotherapy, Programmed death ligand 1, Programmed cell death protein 1, PD-1, PD-L1, Test, Antibody, Diagnostic, Tests

## Abstract

**Background:**

The programmed death receptor 1 (PD-1) protein is a cell-surface receptor on certain lymphocytes that, with its ligand programmed death ligand 1 (PD-L1), helps to down-regulate immune responses. Many cancer types express PD-L1 and evade immune recognition via the PD-1/PD-L1 interaction. Precision therapies targeting the PD-1/PD-L1 pathway have the potential to improve response and thereby offer a novel treatment avenue to some patients with cancer. However, this new therapeutic approach requires reliable methods for identifying patients whose cancers are particularly likely to respond. Therefore, we conducted a systematic literature review assessing evidence on test validation and scoring algorithms for PD-L1 immunohistochemistry (IHC) tests that might be used to select potentially responsive patients with bladder/urothelial cell, lung, gastric, or ovarian cancers for immunotherapy treatment.

**Methods and results:**

To identify evidence on commercially available PD-L1 IHC assays, we systematically searched MEDLINE and Embase for relevant studies published between January 2010 and September 2016 and appraised abstracts from recent oncology conferences (January 2013 to November 2016). Publications that met the predefined inclusion criteria were extracted and key trends summarized.

In total, 26 eligible primary studies were identified, all of which reported on the test validation metrics associated with PD-L1 IHC tests in lung cancer, most using immunohistochemistry testing. There was significant heterogeneity among the available tests for PD-L1. Specifically, no definitive cutoff for PD-L1 positivity was identifiable, with more than one threshold being reported for most antibodies. Studies also differed as to whether they evaluated tumor cells only or tumor cells and tumor-infiltrating immune cells. However, all of the tests developed and validated to support a therapeutic drug in the context of phase 2–3 clinical trials reported more than 90% inter-reader concordance. In contrast, other PD-L1 antibodies identified in the literature reported poorer concordance.

**Conclusions:**

Published validation metric data for PD-L1 tests are mainly focused on immunohistochemistry tests from studies in lung cancer. The variability in test cutoffs and standards for PD-L1 testing suggests that there is presently no standardized approach. This current variability may have implications for the uptake of precision treatments.

## Background

Checkpoint inhibitor therapy is a recent development in the field of cancer immunotherapy and precision medicine, and involves targeting immune pathways that enhance the body’s ability to recognize and destroy tumor cells (TCs). One key mediator in such pathways is the programmed death receptor 1 (PD-1) protein, a cell-surface receptor on certain lymphocytes. The interaction between PD-1 and its ligand, programmed death ligand 1 (PD-L1), plays a crucial regulatory role in the human immune system by inhibiting the body’s immune response to foreign antigens. However, many cancer cell types express PD-L1 and thereby activate PD-1/PD-L1 signaling, thus enabling these tumors to evade immune recognition. Precision therapies that focus on the PD-1/PD-L1 pathway can offer a novel treatment avenue to some patients with cancer. Five PD-1/PD-L1 immunotherapies (atezolizumab, avelumab, durvalumab, nivolumab and pembrolizumab) have now been approved by the United States (US) Food and Drug Administration (FDA) and/or European Medicines Agency (EMA) for a variety of indications following the publication of clinical trials demonstrating their efficacy improving therapeutic response.

Although research into the effectiveness of these types of immunotherapy is rapidly evolving, there remains some uncertainty regarding the extent to which measuring levels of PD-L1 expression in individuals’ tumor tissue helps to identify patients who are most likely to respond to treatment. For example, in Hodgkin’s lymphoma, most tumors have been reported to express PD-L1, so assessing expression in patients can contribute only minimally to clinical decision-making about suitability for treatment [1]. However, for a specific group of cancers (e.g., non-small cell lung cancer), evidence suggests that responsiveness to PD-1 inhibitors such as pembrolizumab and nivolumab or to the anti-PD-L1 antibodies atezolizumab and durvalumab may be predicted by expression of PD-L1 on TCs and/or tumor-infiltrating immune cells (ICs) [1]. Therefore, tests detecting PD-L1 expression may play an important role in the use and development of anti PD-1/PD-L1 agents aimed at these tumor types, which include bladder/urothelial cell, lung, gastric, and ovarian cancer.

Currently there are a range of commercially available PD-L1 IHC tests. Tests are typically designated by the antibody clone that is used to detect the presence of the PD-L1 protein; for example, the 22C3 test developed by Dako (PD-L1 IHC 22C3 pharmDx, Agilent Pathology Solutions) uses a monoclonal mouse anti–PD-L1 clone, 22C3. Some of the available tests have been developed and validated as part of clinical trials that were used to demonstrate the efficacy of the aforementioned licensed PD-1/PD-L1 immunotherapy medicines. Tests of this type can be further sub-divided into two types: companion diagnostics, which (per the US Food and Drug Administration (FDA) definition), provide information, often obtained in vitro, that is “essential for the safe and effective use of a corresponding drug or biologic product” [2], and complementary (or co-diagnostic) tests that may be used in treatment selection, but are not considered essential for safe and effective use of the corresponding therapy in practice. A key distinction between companion and complementary diagnostics is that, whereas companion diagnostics are tied to a specific drug within its approved label, complementary or co-diagnostics may be associated with particular drugs but are not included in the licensing indications for those drugs. Of note, IHC-22C3 for pembrolizumab is currently the only FDA-approved companion diagnostic for PD-1/PD-L1 targeted immunotherapies. Furthermore, although pembrolizumab is now licensed for multiple indications, the FDA only recommends IHC-22C3 for treatment selection for the following specific groups: patients with previously untreated metastatic non-squamous non-small cell lung cancer (NSCLC) whose tumors express PD-L1 at a level of 50% of higher (or second line NSCLC patients with ≥1% expression) and patients with recurrent locally advanced or metastatic, gastric or gastroesophageal junction adenocarcinoma who have Combined Positive Score (CPS) (a measure based on the number of PD-L1 stained tumor cells, lymphocytes, macrophages) of ≥1. Other tests such as IHC 28–8, SP142, and SP263 for nivolumab, atezolizumab and durvalumab respectively, are regarded as complementary diagnostics and are not considered by the FDA as being essential for safe and effective treatment selection.

The landscape of available potential PD-L1 diagnostic tests is further complicated by the fact that each test has its own antibody detection system and tests are performed using different platforms. As a result, the extent to which particular tests are either interchangeable across different indications or superior in terms of accuracy can be important to both uptake of PD-1/PD-L1 targeted therapies and use of these tests for patient management decisions. To provide insights into this area and to help identify and address potential knowledge gaps, a systematic literature review (SLR) was conducted to provide insights into the characteristics of different tests and to examine the validity of commercially available PD-1/PD-L1 tests in assessing bladder/urothelial cell, lung, gastric, and ovarian cancers.

## Objectives

This review explored the characteristics of commercially available PD-L1 tests currently in use for bladder/urothelial cell, lung, gastric, and ovarian cancers, by addressing the following specific research questions:

- What types of tests, platforms, and scoring algorithms are currently being used?
- How has the validity of these tests, platforms, and scoring algorithms been tested?

## Methods

The SLR was conducted in accordance with the methods outlined in the Preferred Reporting Items for Systematic Reviews and Meta-Analyses (PRISMA) guidelines.

Systematic searches were conducted in MEDLINE® (via PubMed) and Embase® (via embase.com) for studies published in English between January 1, 2010 and September 15, 2016. Medical Subject Headings (MeSH), EMTREE terms, and free-text terms were used and combined, where appropriate, with Boolean operators (“AND”, “OR,” and “NOT”). Key search terms included text variations on biomarkers of interest, such as “programmed death-ligand,” “PDL1,” “PD-L1,” and relevant validation metrics, such as “Sensitivity and Specificity” (MeSH) and “valid*.” (The MEDLINE search strategy is provided in a supplementary appendix.) Two searches were run; the second supplementary search used the same core algorithm but with some additional terms (for example “correlat*” and “immunohistochemistry” [MeSH]) to ensure the search was comprehensive.

Supplementary searches were undertaken to capture ‘grey’ literature—data from sources not indexed in the electronic databases. To capture such evidence, proceedings from the three most recent meetings of the following six subject-specific conferences were searched:

1. American Society of Clinical Oncology (ASCO)
2. European Society for Medical Oncology (ESMO)
3. Society for Immunotherapy of Cancer (SITC)
4. International Cancer Immunotherapy Conference
5. American Association of Cancer Research (AACR)
6. International Association for the Study of Lung Cancer (IASLC)

Study selection was based on criteria that were defined a priori and are summarized in Table 1. The titles and abstracts of records retrieved via the literature searches were first appraised by a single reviewer, and 10% of the screening decisions made at this level were checked by second reviewer to confirm their accuracy, as a quality control measure. Relevant studies that passed this first round of screening then underwent full-text screening, which was conducted by two reviewers to confirm each inclusion and exclusion decision. Any discrepancies at the abstract and full-text level were resolved in discussion with a third reviewer where necessary.

**Table 1:** Criteria for Study Selection

Criteria	Inclusion Criteria	Exclusion Criteria	Rationale
Population(s)	Patients with bladder/urothelial cell, lung, gastric, or ovarian cancer	• Ongoing studies • Interim analyses • Studies of other oncology indications	Population criteria were designed to reflect cancer populations that are candidates for PD-L1 expression testing
Interventions/Comparators	Diagnostic tests targeting the PD-1/PD-L1 pathway	N/A	To survey the range of tests currently in use, all PD-L1 tests or studies looking at diagnostics used in PD-1/PD-L1 immunotherapy trials were considered
Outcomes	PD-L1 test-validation metrics. Information on PD-L1 test-scoring algorithms or cutoffs was also captured from those studies that reported on test performance	Studies that did not report outcomes of interest for the study population	As the review aimed to evaluate how well different tests performed against validation criteria, studies reporting outcomes relating to validation metrics were prioritized. It was also considered important to capture data relating to the tests’ characteristics (scoring algorithms and test cutoffs) in order to determine the comparability of different tests
Time	Indexed databases: January 1 2010 to September 15, 2016) Grey literature: Three most recent meetings (January 2013 up to November 2016).	Studies published prior to 2010 or after the final search date in 2016	Date limits were applied to reflect the very recent/current nature of this field of research
Study Design	• Randomized trials • Observational studies • Diagnostic or clinical validation studies	• Animal studies • Case reports • Editorials	Study design criteria reflected the nature of the studies reporting on test-validation metrics of PD-L1 tests for use in human population.
Other	PD-L1 tests required to be commercially available • English language only • Geographic emphasis on the US, EU5, and Japan	• Articles that were either not published in English or outside the geographic locations of interest • Publications on noncommercially available tests	Commercially available tests were prioritized to ensure that review was relevant to current practice. The geographic emphasis reflects the countries in which PD-1/PD-L1 immunotherapies are currently licensed. Most evidence in this field is published in English so language limits were designed to reflect this.

*Abbreviations*: *EU5* European Union 5, *N/A* not applicable, *PD-1* programmed death receptor 1, *PD-L1*, programmed death ligand 1, *US* United States

Data abstraction of the included studies was performed using a predefined data abstraction template designed in Microsoft Excel®. For each included study, data were captured by a single investigator, with validation of the accuracy and completeness of this abstraction being performed by a second reviewer. Any discrepancies were resolved in a discussion with a third investigator. Specific key information was abstracted from included studies on the following: patient population, type of test, test developer, test platform, test-scoring algorithms, test thresholds/cutoffs, and test-validation metrics. Due to the variety of study designs considered in this review, it was not possible to undertake a risk-of-bias assessment using a single standardized tool. Heterogeneity in the studies also meant that a quantitative meta-analysis of their data was not appropriate; therefore, the evidence abstracted from included studies was qualitatively synthesized and key trends were summarized.

## Results

### Search results

The indexed database searches yielded 950 records. After removing publications duplicated between databases, 589 abstracts remained and were screened, of which 57 met the criteria for detailed review of their associated full-text publications. Of these 57 publications subjected to full-text screening, 12 were eligible for inclusion in the SLR, as they reported on PD-L1 test validation metrics for commercially available tests. An additional eight studies were identified from the supplementary search and 10 conference abstracts also met the eligibility criteria. Therefore, a total of 30 references (collectively representing 26 unique study populations and four linked publications) were included in the review. The study screening and selection process is illustrated in Fig. 1.

**Fig. 1:** Screening and Study Selection

All 26 included studies reported on test validation metrics associated with PD-L1 tests in lung cancer. One of the studies also reported data relating to bladder/urothelial cell cancer [3]. No evidence relating to gastric or ovarian cancer was identified.

### Lung cancer

#### Types of PD-L1 antibody tests identified in the SLR

Across the 26 included studies, eight antibodies for detecting PD-L1 expression in patients with lung cancer were identified, as follows:

- PD-L1 IHC 22C3 pharmDx by Dako (referred to hereafter by the antibody 22C3): 3 studies [4–6]
- PD-L1 IHC 28–8 pharmDx by Dako (referred to hereafter by the antibody 28–8): 7 studies [6–12]
- VENTANA PD-L1 (SP263) Rabbit Monoclonal Primary Antibody by Roche (referred to hereafter by the antibody SP263): 6 studies [6–8, 13–15]
- VENTANA PD-L1 (SP142) Assay by Roche (referred to hereafter by the antibody SP142): 9 studies [3, 6, 8, 9, 16–20]
- PD-L1 (E1L3N®) XP® Rabbit mAb #13684 by Cell Signaling Technology [CST] (a reagent provider): 9 studies [8, 11, 15, 20–25]
- 4059 by ProSci, Inc.: 1 study [26]
- h5H1 by Advanced Cell Diagnostics: 1 study [27]
- 9A11 (developer not reported): 1 study [8]

In all cases, PD-L1 expression was evaluated using an immunohistochemistry (IHC) platform. One of the studies specified that diaminobenzidine tetrahydrochloride was used as the reagent to produce the “brown staining” for the IHC process [8]. Three studies evaluated results derived from alternative test platforms as well as IHC. Two studies [8, 20] measured PD-L1 expression using quantitative fluorescence (QIF) and another study looked at fluorescence in-situ hybridization (FISH) [12].

The antibodies manufactured by Dako and Roche had all been originally developed and validated to support a therapeutic drug in the context of a clinical trial. These antibodies were evaluated in eight studies as follows:

- Three studies looked at the IHC-SP142 (Roche), developed alongside atezolizumab [3, 16, 17]
- Two studies looked at IHC-SP263 (Roche), developed alongside durvalumab [14, 28]
- Two studies looked at IHC-22C3 (Dako), developed alongside pembrolizumab [4, 5]
- One study looked at IHC-28-8 (Dako), developed alongside nivolumab [10]

#### Test-scoring algorithms and thresholds used among the PD-L1 tests

The thresholds and scoring systems used to determine PD-L1 positivity varied between the antibodies and across studies. Eleven studies [4, 7, 10–12, 14, 19–21, 23, 28] investigated dichotomous cutoffs (representing the proportion of cells with PD-L1 expressed) for PD-L1 positivity using different antibodies (the thresholds used in these studies are summarized in Table 2). Amongst these 11 studies, nine [4, 6, 9–11, 19, 20, 22, 27] set thresholds a priori (for example, based on cutoffs used in previously published research) and two studies [4, 13] attempted to establish an optimal threshold based on the study findings. In one study [18], it was unclear whether the thresholds used had been specified prospectively or retrospectively.

**Table 2:** Dichotomous Scoring Used Across Antibodies for PD-L1 IHC Tests in Lung Cancer

Antibody (developer) [drug against which the study validated the test]	Cutoff/Threshold
22C3 (Dako) [pembrolizumab]	1% (used in training group): 1 study [4]^a^ 50% (determined as optimal cutoff): 1 study [4]^a^
28–8 (Dako) [nivolumab]	1%: 3 studies [7, 10, 12]^a^ 5%: 2 studies [10, 11]^a^ 10%: 1 study [10]^a^ 50%: 1 study [11]^a^
SP263 (Roche) [durvalumab]	25%: 3 studies [7, 14, 28]^a,b^
SP142 (Roche) [atezolizumab]	1%: 2 studies [19, 20]^a^ 5%: 2 studies [19, 20]^a,c^ 50%: 1 study [20]^a^
E1L3N (Cell Signaling Technology; reagent provider) [not applicable]	1%: 2 studies [20, 21]^a^ 5%: 4 studies [11, 20, 21, 23]^a,c^ 50%: 3 studies [11, 20, 21]^a^

^a^Tested in tumor cells. ^b^ Tested in tumor-infiltrating immune cells. ^c^ Tested in tumor stroma

A further 11 studies [5, 9, 13, 15–17, 22, 24–27] used a hybrid score that combined components of staining intensity with the percentage of positive cells to determine PD-L1 positivity. One study evaluated two tests, SP142 (Roche) and E1L3N (CST; reagent provider), by means of a QIF process that used an automated scoring system. In this system, the QIF score of PD-L1 signal for each antibody in the tumor and stroma was calculated by dividing the target PD-L1 pixel intensities by cytokeratin and DAPI positivity [20].

A second study [8] that incorporated QIF did not provide details on the scoring approach. Another study [12] investigated FISH and evaluation criteria included CD274, PDCDILG2-CEB 9 ratio, gene copy numbers, proportions of TCs with ≥4 PDL1/2 and ≥5 PDL1/2 signals, and gene clusters. Yet another study [6] validated a six-step scoring system that integrated all of the cutoff criteria from four tests that have been used in clinical trials: 28–8 and 22C3 (both Dako) and SP142 and SP263 (both Roche).

#### Types of cells tested for PD-L1 expression

There was variation among the studies with regard to the cell type tested, specifically, whether PD-L1 expression was measured on TCs and/or tumor-infiltrating ICs. Nine studies tested TCs only [4, 5, 7, 10–12, 21, 26, 27], two tested both TCs and tumor stroma [20, 29], 14 studies evaluated both TCs and ICs [3, 6, 8, 9, 13–17, 19, 22, 24, 25, 28], and in one study it was unclear which type of cell had been tested [23]. TCs were more frequently evaluated than tumor-infiltrating ICs or tumor stroma, regardless of whether dichotomous or hybrid scoring algorithms were used.

#### Test validation metrics

##### Individual test performance

Most studies (18/26) focused on a single antibody and reported validation metrics that were specific to the one test under investigation, without comparing its performance with that of another antibody or testing approach. The results of these studies by outcome are summarized below and in Table 3. Among the tests developed in a clinical trial setting to accompany a therapeutic product, the validation metrics were similar and all the tests had a greater than 90% inter-observer concordance [10]. In comparison, E1L3N, a test developed outside of clinical-trial settings [i.e., not specifically for a particular PD-1/PD-L1–targeted therapy], reportedly had slightly lower inter-observer concordance metrics [21–23], namely below the 84–88% concordance level at the 1% cutoff [21]. In the studies that reported intra-observer and inter−/intra-site concordance, high agreement (above 90%) was observed for all these metrics across the tests developed in a clinical trial setting to accompany a therapeutic product, except for inter-site concordance for SP263 (Roche; durvalumab), which was 86.4% [14] and for 22C3 (Dako; pembrolizumab) 88.3% [5].

**Table 3:** Individual Test Performance: Test-Concordance Metrics

Study Information	Inter-Observer Concordance % (95% CI)	Intra-Observer Concordance % (95% CI)	Inter-Site Concordance % (95% CI)	Intra-Site Concordance % (95% CI)
Antibody (developer): 22C3 (Dako) Roach et al. (2016) [Trial name: KEYNOTE-001] [5] Indication: NSCLC Drug against which the study validated the test: pembrolizumab	**ANA**: 92.6% (87.8%–96.7%) **APA**: 92.8% (88.1%–96.8%) **OA**: 92.7% (88.1–96.8%)	**ANA**: 96.4% (94.0%–98.5%) **APA**: 96.5% (94.3%–98.6%) **OA**: 96.4% (94.3%–98.6%)	**ANA**: 90.3% (84.4%–95.2%) **APA**: 85.2% (75.6%–92.9%) **OA**: 88.3% (81.4%–94.3%)	**ANA**: 91.9% (88.8%–94.8%) **APA**: 87.6% (82.5%–92.2%) **OA**: 90.2% (86.3%–93.7%)
Antibody (developer): 28–8 (Dako) Phillips et al. (2015) [10] Indication: NSCLC Drug against which the study validated the test: nivolumab	1% Cutoff **ANA**: 96.1% (94.7%–97.4%) **APA**: 96.5% (95.2%–97.7%) **OA**: 96.3% (94.9%–97.5%) 5% Cutoff **ANA**: 91.3% (89.2%–93.2%) **APA**: 89.3% (86.8%–91.6%) **OA**: 90.4% (88.3%–92.3%)	1% Cutoff **ANA**: 97.7% (95.6%–99.3%) **APA**: 97.9% (96.0%–99.3%) **OA**: 97.8% (95.9%–99.3%) 5% Cutoff **ANA**: 98.7% (97.2%–99.7%) **APA**: 98.3% (96.5%–99.6%) **OA**: 98.5% (97.0%–99.6%)	1% Cutoff **ANA**: 93.9% (92.4%–95.3%) **APA**: 95.5% (94.4%–96.5%) **OA**: 94.8% (93.6%–95.9%) 5% Cutoff **ANA**: 90.2% (88.5%–91.8%) **APA**: 90.2% (88.5%–91.8%) **OA**: 90.2% (88.6%–91.8%)	1% Cutoff **ANA**: 97.0% (95.2%–98.4%) **APA**: 97.7% (96.5%–98.9%) **OA**: 97.4% (95.9%–98.7%) 5% Cutoff **ANA**: 94.8% (92.8%–96.7%) **APA**: 94.8% (92.8%–96.7%) **OA**: 94.8% (92.8%–96.7%)
Antibody (developer): SP263 (Roche) Rebelatto et al. (2016) [14] Indication: NSCLC Drug against which the study validated the test: durvalumab	**APA**: 96.6% (93.8%–98.8%) **ANA**: 96.8% (93.9%–98.9%) **OPA**: 96.7% (94.2%–98.9%)	**APA**: 96.2% (92.7%–98.8%) **ANA**: 96.4% (93.0%–98.8%) **OPA**: 96.3% (93.3%–98.8%)	**PPA**: 93.3% (89.0%–95.9%) **NPA**: 79.5% (73.6%–84.4%) **OPA**: 86.4% (82.7%–89.3%)	NR
Antibody (developer): SP142 (Roche) Boyd et al. (2015) [3] Indication: NSCLC Drug against which the study validated the test: atezolizumab	Met predefined acceptance criteria including > 90% inter-reader concordance.	NR	NR	NR
Antibody (developer): E1L3N (CST^a^) Gainor et al. 2016 [21] Indication: NSCLC (EGFR-mutant and ALK-positive) Drug against which the study validated the test: PD-1/PD-L1 inhibitors	Concordance between the two pathologists: 1%: 0.88 (κ = 0.75) 5%: 0.92 (κ = 0.80) 50%: 0.97 (κ = 0.89)	NR	NR	NR
Antibody (developer): E1L3N (CST^a^) Inamura et al. (2016) [23] Indication: lung (adenocarcinoma, surgically resected) Drug against which the study validated the test: N/A	Agreement between two pathologists: 5%: κ = 0.70 (95% CI 0.55–0.86), indicating substantial agreement	NR	NR	NR
Antibody (developer): E1L3N (CST^a^) Huynh et al. (2016) [22] Indication: lung (adenocarcinoma, surgically resected) Drug against which the study validated the test: N/A	Agreement between two pathologists: 1%: 0.84 (κ = 0.69) 5%: 0.91 (κ = 0.81) 50%: 0.91 (κ = 0.78)	NR	NR	NR

^a^CST is a reagent provider

*Abbreviations*: *ALK* anaplastic lymphoma kinase, *ANA* negative percent agreement, *APA* positive percent agreement, *CST* Cell Signaling Technology, *EGFR* epidermal growth factor receptor, *N/A* not applicable,, *NR* not reported, *NSCLC* non-small cell lung cancer, *OA* overall agreement, *OPA* Overall Percentage Agreement, *PD-1* programmed death receptor 1, *PD-L1* programmed death ligand 1, *PPA* positive percent agreement

Two studies reported on the extent of agreement in test results when different types of samples (biopsy or surgical-resection) were tested, and these found some conflicting results. One study looked at the use of the SP142 test (Roche) in biopsy and surgical-resection samples. It reported an overall discordance rate of 48% (95% confidence interval, 4.64%–13.24%) and a κ score of 0.218, indicating poor agreement between the test outputs from the different sample types [13]. The study authors commented also that in all cases, the biopsy specimens underestimated the PD-L1 status relative to the expression level in the whole tumor (further data not provided in the study report). Another study found overall concordance between biopsy and surgical-resection samples ranged from 82.5% (κ = 0.3969) (i.e., fair agreement), at a score of hybrid score of 51 (range, 0–170) or greater, to 92.4% (κ = 0.8366) (i.e., high agreement), at a score of 1 or greater [26].

##### Head-to-head test performance

Seven studies reported data relating to the comparative performance of two or more tests, and their key findings are summarized in Table 4. Among these studies, three reported on the overall test concordance between two or more antibodies. The first found acceptable agreement between two tests developed in a clinical trial setting to accompany a therapeutic product, 28–8 (Dako; nivolumab) and SP263 (Roche; durvalumab), for which the overall test concordance was 90.3%. The remaining two studies found mixed results when a clinical trial test developed to support a therapeutic product was compared with E1L3N, which was not developed or validated as part of a clinical trial. Of these studies, one observed poor concordance when SP142 (Roche, atezolizumab) was compared with the antibody E1L3N (CST; reagent provider, not developed or validated as part of a clinical trial) (κ concordance at 1% cutoff = 0.340, 5% cutoff = 0.286, and 50% = 0.189) [20]. The other study reported moderate agreement between 28 and 8 (Dako, nivolumab) and E1L3N (75.0% and 86.2% at 5% and 50% cutoffs, respectively) [11].

**Table 4:** Head-to-Head Test Performance: Test-Validation Metrics

Study Information	Type of Test (developer)	Overall Concordance/Discordance Between Tests	Other Comparisons Between Tests	Authors’ Conclusions
Anderson et al. (2016) [7] Drug against which the study validated the test: N/A	28–8 (Dako) and SP263 (Roche)	Overall concordance between antibodies was 90.3%, but was only 66.7% for specimens considered positive for PD-L1 expression	There was considerable variation in the percentage of TC staining positive as determined by the two methods, which along with the different test cutoffs contributed to discordant results	This study points to the importance of methodological and interpretation variation, as well as other considerations such as tumor heterogeneity and dynamics of expression, when evaluating the use of PD-L1 as a biomarker of potential therapeutic response to checkpoint blockade inhibitors
McLaughlin et al. (2016) [20] Drug against which the study validated the test: N/A	E1L3N (CST^a^) and SP142 (Roche)	PD-L1 Comparison Using Different PD-L1 Antibodies and IHC κ concordance between antibodies was low, irrespective of the cutoff used: • 1% tumor PD-L1 cutoff: 0.340 • 5% tumor PD-L1 cutoff: 0.286 • 5% stroma PD-L1 cutoff: 0.124 • 50% tumor PD-L1 cutoff: 0.189		Concordance between the two rigorously validated antibodies was fair to poor.While both E1L3N and SP142 reportedly bind to the intracellular domain of PD-L1, the difference between the two antibodies raises concerns and suggests antibody-validation data should be shown in future clinical trial reports
Rivalland et al. (2016) [11] Drug against which the study validated the test: N/A	E1L3N (CST^**a**^) and 28–8 (Dako)	The concordance between antibodies was 75.0% and 86.2% at 5% and 50% cutoffs, respectively	• E1L3N stained a significantly higher proportion of tumors at both cutoffs (*P* < 0.001), and in almost all clinic-pathologic subgroups • A significant correlation was observed in staining between antibodies (R^2^ = 0.40, *P* < 0.0001) • Small-cell lung cancer stained significantly more frequently than adenocarcinoma with Dako 288 (35.7% vs. 17.4%, *P* < 0.001) but not with E1L3N (44% vs. 35.1%, *P* < 0.08)	Overall PD-L1 positivity was correlated between these two antibodies, however the CST^a^ antibody stained significantly more samples
Scheel et al. (2016) [6] Drug against which the study validated the test: N/A	28–8, 22C3, SP142, and SP263 (NR)	• NR	• The tests 28–8 and 22C3 stained comparable TC proportions • In some cases, SP142 stained fewer TCs but more ICs and SP263 stained more TCs and ICs compared with the other tests • The differences in TC proportions would translate into different classifications by any of the dichotomous cutoffs	• The data indicate that unified PD-L1 IHC scoring criteria for TCs are feasible, while scoring of ICs requires detailed training • The four tested PD-L1 tests did not show comparable staining patterns in all cases of NSCLC • The results obtained by each test are not interchangeable. Thus, more studies are required to archive a harmonized “PD-L1 status” in NSCLC • In particular, more data on the predictive value of one test for multiple substances are needed
Smith et al. (2016) [15] Drug against which the study validated the test: N/A	SP263 (Roche) and E1L3N (CST^a^)	NR	Inter-pathologist correlation Membrane tumor staining scores • SP263: R^2^ > 0.87 • E1L3N: R^2^ > 0.82 Positively staining cells in the immune infiltrate • SP263: R^2^ > 0.66 • E1L3N: R^2^ > 0.80	Due to its staining intensity, scoring range, and pathologist preference, the SP263 IHC test has been deemed superior to the E1L3N IHC test
Ilie et al. (2016a) [13] Drug against which the study validated the test: N/A	SP142 and SP263 (Roche); and 28–8 (Antibodycam)	Inter-reader precision in determining the PD-L1 expression in TCs: • OA: 92% (κ = 0.910), 98% (κ = 0.976) and 96% (κ = 0.935) for SP142, SP263 and 28–8 tests Inter-reader precision in determining the PD-L1 expression in ICs: • OA: 81% (κ = 0.786), 87% (κ = 0.832), and 86% (κ = 0.817) for SP142, SP263 and 28–8 tests, respectively	Concordance analysis on TCs: • Poor correlation between the SP142 and SP263 antibodies (ρ = 0.852, κ = 0.362), and the SP142 and 28–8 antibodies (ρ = 0.860, κ = 0.412), while a good correlation was observed between the SP263 and 28–8 antibodies (ρ = 0.996, κ = 0.883) Concordance analysis on ICs: • Poor agreement between the SP142 and SP263 antibodies (ρ = 0.568, κ = 0.018) and the SP142 and 28–8 antibodies (ρ = 0.590, κ = 0.134), while a good correlation was noted between the SP263 and 28–8 antibodies (ρ = 0.880, κ = 0.721)	Our results suggest that PD-L1 protein expression is heterogeneous and that different antibody tests may yield variable results. The anti-PD-L1 antibodies SP142 vs. SP263, and SP142 vs. 28–8 showed fair to poor concordance, while the 28–8 and SP263 antibodies demonstrated a strong correlation for both the TC and IC compartments
Schildhaus et al. (2016) [1**2]** Drug against which the study validated the test: N/A	IHC: 28–8 (Dako) and FISH: ZytoLight SPEC CD274, PDCDILG2/CEN 9 Dual Color Probe	The correlation between IHC and FISH was statistically significant (χ^2^: *P* < 0.001)	NR	PD-L1/2 FISH could contribute to our understanding of PD-L1 expression and could therefore be a valuable adjunct biomarker in upcoming trials with PD-1/PD-L1 inhibitors

^a^CST is a reagent provider

*Abbreviations*: *CST* Cell Signaling Technology, *FISH* fluorescence in-situ hybridization, *IC* immune cell, *IHC* immunohistochemistry, *N/A* not applicable, *NR* not reported, *NSCLC* non-small cell lung cancer, *OA* overall agreement, *PD-1* programmed death receptor 1, *PD-L1* programmed death ligand 1, *TC* tumor cell

Three of the head-to-head comparison studies [6, 13, 15] reported on differences between TC and IC staining patterns between antibodies, and they found mixed results: in some cases, SP142 stained fewer TCs but more ICs, whereas SP263 stained more TCs than ICs [6]. A further study [13] found good overall concordance between the SP142 and SP263 (both Roche) antibodies on TCs (κ = 0.412) but poor agreement between these antibodies on ICs (κ = 0.018). This study also reported poor agreement between SP142 and 28–8 antibodies [13] on TCs (κ = 0.412) and ICs (κ = 0.134), whereas good concordance was observed between the SP263 and 28–8 antibodies on both TCs (ρ = 0.996, κ = 0.883) and ICs (κ = 0.721). Another study [15] compared SP263 (Roche) with E1L3N (CST; reagent provider) and found that inter-pathologist correlation for membrane-tumor staining was similar between the antibodies (SP263 R2 > 0.87 vs E1L3N R2 > 0.82), while staining for ICs was lower with SP263 (R2 > 0.66) than with E1L3N (R2 > 0.80).

##### Harmonization of scoring algorithms across antibodies

One study reported on inter-observer concordance based upon a six-step scoring system which integrated the criteria employed by the four different clinical trial tests (28–8 and 22C3 [both Dako], SP142 and SP263 [both Roche]) and found moderate agreement using this harmonized approach (κ = 0.47 to 0.49) [6]. The study also reported good concordance coefficients (κ = 0.59 to 0.80) when using integrated dichotomous proportion cutoffs across the antibodies (≥ 1%, ≥ 5%, ≥ 10%, ≥ 50%); however, proportion scoring of PD-L1–positive IC yielded lower inter-observer concordance coefficients both for the six-step score (κ < 0.2) and the dichotomous cutoffs (κ = 0.12 to 0.25), concluding that unified PD-L1 IHC scoring criteria for TCs may be feasible, whereas scoring for ICs requires detailed training [6].

### Bladder cancer

One study reported on the test-validation performance of a PD-L1 test in bladder/urothelial cell cancer for the antibody SP142 (Roche) and found it had acceptable inter-reader concordance between pathologists (> 90%) when measuring PD-L1 expression in both IC and TC in bladder/urothelial cell cancer [3].

## Discussion

The results of this SLR demonstrate that there are varied cutoff and scoring algorithm approaches among the commercially available PD-L1 antibody tests in lung cancer. There is, for example, no commonly accepted standard or threshold for determining positivity for each of the antibodies based on the proportion of PD-L1–positive cells. Further differences between scoring algorithms relate to the way in which staining patterns are interpreted; some studies have investigated the use of proportional scoring [4, 7, 10–12, 14, 19–21, 23, 28] for the respective antibodies, whereas other studies have looked at hybrid test-scoring methods that also take into account staining intensity [5, 13, 15–18, 22, 24–27].

In general, our review found that the concordance between tests developed in a clinical trial setting to accompany a therapeutic product was deemed acceptable, with inter-reader concordance exceeding 90% [7]. This finding is mirrored in recently published data from phase 1 of the Blueprint Project, which explored the analytical and clinical comparability of four PD-L1 IHC tests used in clinical trials (Dako 22C3, Dako 28–8, Roche SP142, and Roche SP263) and found comparable results across the tests when applied to assess TC staining in NSCLC, although the test SP142 resulted in fewer stained TCs overall (phase 2 of this project is now underway and will seek to validate these findings and also provide data on a fifth assay developed by Dako that uses the antibody 73–10). Our SLR did, however, find conflicting evidence concerning concordance when different antibodies developed in a clinical trial setting to accompany a therapeutic product were compared with those developed outside this type of setting, such as E1L3N [11, 15, 20].

Our findings are in line with other reviews in this topic area (which were performed non-systematically), which have also reported on the variations in cutoffs used for different antibodies to determine PD-L1 positivity [30–32]. In particular, our research did not identify a definitive threshold result that can be universally applied to predict clinical response to PD-L1–targeted precision treatments, which has been noted previously by Festino et al. [30]. There were also differences among the studies included in our review in terms of the types of cells that were tested for PD-L1 expression (i.e., TCs only, or TCs and ICs), with some studies [13, 15] also noting differences in staining patterns and concordance depending on whether biopsy and surgical resection samples were tested. Two recent review articles have also reported that cell type can play a key role in determining test outcomes. Specifically, these publications have indicated that ICs express significantly higher levels of PD-L1 than TCs (e.g., Ma et al. [31] and Festino et al. [30]) and that the expression by TCs is sometimes more heterogeneous compared with that of ICs. It has also been theorized that different cell phenotypes/characteristics may also contribute to this variability in PD-L1 expression across cancer cells [32].

One limitation of our review is that of the existing commercially marketed tests considered, most were IHC tests, with only three studies reporting on QIF [8, 20] and FISH [12]. We did not, for example, find any data on multimarker or next-generation tests that identify PD-L1 expression. In addition, only limited evidence was found on PD-L1 tests in bladder/urothelial cell cancer, and there were no validation studies for commercially available tests in gastric or ovarian cancers.

The heterogeneity in the findings of this review has important implications for clinical practice. Notably, the lack of standard thresholds for responder identification and concordance between a subset of tests indicates the existence of (1) potential risks for efficient treatment selection and use of precision therapies; (2) confusion about whether it is important to request a particular PD-L1 test; and (3) potential adverse effects on patient management decisions (e.g., if the test thresholds used in clinical practice do not correspond with those used in the clinical trials in which particular IHC clones were developed and validated, and in which treatment efficacy was demonstrated, the patient may be inaccurately identified as a potential therapy recipient). However, it is also important to note that no study from our search results reported evidence for these possibilities. Ambiguity around test thresholds, decision algorithms, and interchangeability of PD-1/PD-L1 testing could also present uncertainty for those payers who view accurate prediction of the subpopulation of treatment responders as being a key value of precision therapy approaches. Where there is variability in the interpretation or selection of particular tests, there is the potential for physician confusion, interpretation dilemmas, and payer uncertainty.

There are illustrative examples of such difficulties from previous attempts to introduce biomarker testing to the selection of precision therapy and patient management. In the case of IHC and molecular testing for epidermal growth factor receptors, for instance, the substantial variability in test cutoffs or thresholds and the potential for variable interpretation of early-generation tests have been well documented. Following early introduction of tests for this marker and initial launch of EGFR-targeted agents, some health technology assessment and payer organizations (notably, large commercial health plans in the United States and the Canadian Agency for Drugs and Technologies in Health [33] in Canada) had concerns around interpretation and selection of some EGFR tests, arguing that the connection between test results and patient management or treatment selection was insufficiently clear. Another example occurred in the years immediately following the launch of trastuzumab, when there was significant controversy among physicians over the selection of HER2 IHC vs. FISH testing that led, in some cases, to slower uptake of the associated precision medicines. When clinical practice guidelines were updated to indicate that IHC testing should be conducted initially, with a subset of these patients receiving receiving FISH testing for confirmation, this clarified the appropriate clinical testing pathway for prescribing trastuzumab [34]. These instances of uncertainty about how companion diagnostic tests should be interpreted and used had implications for access to precision treatments in some markets, and/or influenced uptake and use of these medicines and their associated tests [34–36].

Conducting additional studies and increasing both interpretation and education about test cutoffs would help to better inform the use of PD-1/PD-L1 diagnostics and ensure more consistent clinical assessment and application of the class of PD-1/PD-L1 inhibitors [31]. In addition, the available literature suggests that greater understanding is needed on the interchangeability of these PD-L1 tests for predicting response to anti-PD-L1 and anti-PD-1 targeted therapies. Such evidence would be crucial for supporting decision-making in a context where multiple PD-L1 tests are available (which seem to have variable validity in inter/intra-observer and inter/intra-site concordance) and where findings are not always consistent or reproducible across tests.

## Conclusions

Most validation-metric data available for PD-L1 tests relate to the use of IHC tests in the context of lung cancer, and this evidence raises some key challenges that may influence the uptake of PD-L1 testing. In particular, standardization among available PD-L1 IHC tests is currently lacking (with regard to antibodies used, cutoffs/thresholds for a given antibody, and differences in scoring algorithm and test sites) and there is limited information on the extent, if any, to which the tests might be interchangeable. Developing strategies to address this variability in available IHC tests and publishing data that clarify the value of non–IHC-based approaches, such as FISH and next-generation tests that incorporate PD-L1, will be important to address as the availability of precision treatments focused on these biomarkers continues to increase.

## Abbreviations

CST: Cell Signaling Technology
IC: Tumor-infiltrating immune cell
IHC: Immunohistochemistry
PD-1: Programmed death receptor 1
PD-L1: Programmed death ligand 1
QIF: Quantitative fluorescence
SLR: Systematic literature review
TC: Tumor cell
